The article "Impact of Single and Stacked Insect-Resistant Bt-Cotton on the Honey Bee and Silkworm" was published in 2013. Journal: PLoS One.

# Impact of Single and Stacked Insect-Resistant Bt-Cotton on the Honey Bee and Silkworm

**DOI:** 10.1371/journal.pone.0072988

**Published:** 2013-09-09

**Authors:** Lin Niu, Yan Ma, Amani Mannakkara, Yao Zhao, Weihua Ma, Chaoliang Lei, Lizhen Chen

**Affiliations:** 1 Hubei Insect Resources Utilization and Sustainable Pest Management Key Laboratory, Huazhong Agricultural University, Wuhan, Hubei, China; 2 Institute of Cotton Research, Chinese Academy of Agricultural Sciences, Anyang, Henan, China; 3 Department of Agricultural Biology, Faculty of Agriculture, University of Ruhuna, Kamburupitiya, Sri Lanka; 4 College of Plant Science and Technology, Huazhong Agricultural University, Wuhan, Hubei, China; French National Institute for Agricultural Research (INRA), France

## Abstract

Transgenic insect-resistant cotton (Bt cotton) has been extensively planted in China, but its effects on non-targeted insect species such as the economically important honey bee (*Apis mellifera*) and silkworm (*Bombyx mori*) currently are unknown. In this study, pollen from two Bt cotton cultivars, one expressing Cry1Ac/EPSPS and the other expressing Cry1Ac/Cry2Ab, were used to evaluate the effects of Bt cotton on adult honey bees and silkworm larvae. Laboratory feeding studies showed no adverse effects on the survival, cumulative consumption, and total hemocyte count (THC) of *A. mellifera* fed with Bt pollen for 7 days. No effects on the survival or development of *B. mori* larvae were observed either. A marginally significant difference between Cry1Ac/Cry2Ab cotton and the conventional cotton on the THC of the 3^rd^ day of 5^th^ *B. mori* instar larvae was observed only at the two highest pollen densities (approximately 900 and 8000 grains/cm^2^), which are much higher than the pollen deposition that occurs under normal field conditions. The results of this study show that pollen of the tested Bt cotton varieties carried no lethal or sublethal risk for *A. mellifera,* and the risk for *B. mori* was negligible.

## Introduction

China is one of the countries taking the lead in planting genetically modified (GM) crops, ranking sixth in the world by 2012 [1]. The planting area of transgenic Bt (*Bacillus thuringiensis* toxin) cotton reached 4.0 million hectares in China in 2012 [1]. Planting of Bt cotton cultivars has proven beneficial because of lower insecticide use and less damage from *Helicoverpa armigera*, the major pest of cotton [2], [3]. An important technique in plant biotechnology is the stacking of resistance to multiple insects or of insect and herbicide resistance traits within a single cultivar [4]. Two new cotton varieties, Cry1Ac/Cry2Ab (both Bt toxins) and Cry1Ac/EPSPS (Bt toxin and 5-enolpyruvyl-shikimate-3-phosphate synthase), were developed in recent years, and they will be commercially available in the foreseeable future in China [5], [6]. The Bt toxins (Cry1Ac and Cry2Ab) target lepidopteran pests [7], [8], and the EPSPS gene makes the plants tolerant to the herbicide glyphosate [9], [10].

Despite the benefits offered by GM plants, they also may have a negative impact on biodiversity and non-target organisms [11]. Thus, laboratory and extended lab/semi-field and field studies are necessary to assess such risks before commercialization [12]. As the first step of assessment of Bt cotton, laboratory tests need to be conducted to evaluate the risks of new cotton varieties on non-target organisms [13].

More than one-third of crops are pollinated by insects and other animals, among which honey bees account for about 80% of the total pollinating insects [14]. A recent study estimated the economic value of honey bee pollination for Chinese agriculture to be worth ¥304.2 billion per year [15]. The honey bee *Apis mellifera* is the most important pollinator species around the world [16], with populations present in all countries growing GM crops [4], [17], including Bt cotton [18]. Pollen is the sole protein source of *A. mellifera* colonies [19], and pollen of many important crops, including cotton [20], is collected by foraging bees [21]. Adults and larvae of *A. mellifera* are directly exposed to transgenic material via pollen consumption of GM crops, which are planted in mass monocultures [13].

The culture of the silkworm *Bombyx mori* is an important export industry that provides considerable income for people in many temperate Asian countries [22]. However, *B. mori* is susceptible to Cry1Ac and Cry2Ab proteins. The larvae of *B. mori* are fed entirely on mulberry leaves, and mulberry plants are often planted near or around the edges of cotton fields. Thus, the larvae may be exposed to the Bt insecticidal proteins expressed in Bt cotton pollen if the pollen is deposited on mulberry leaves [23].

As two economically important insects in China, *A. mellifera* and *B. mori* are key species to be tested for the potential adverse impacts of Bt cotton [18], [23]. To date, few studies have assessed the potential negative impacts of Bt cotton on *A. mellifera* [18], [20], [24], [25] and *B. mori* [23]. Existing results show that Bt toxins have no lethal effect on the two insects. Few studies of the sublethal effects of Bt toxins on *A. mellifera* [18], [20], [26], [27] and *B. mori* [22], [23], [28] have been conducted either. However, as well as the side effects of pesticides on beneficial arthropods [29]–[31], the sublethal effects of Bt toxins on these two economically important insects might negatively impact larval development and immune capacity and lead to colony population decrease [31]. Thus, it is important to evaluate the sublethal effects of transgenic crops on honey bees and silkworms [22], [32], [33].

In China, the flowering period of cotton usually lasts from June to late August, a season during which honey bees have few available floral sources other than cotton. This period is also the time when silkworm rearing occurs [34]. Han et al. demonstrated that another Bt cotton (CCRI41) pollen exhibited highly variable expression of Cry1Ac throughout the season [18], [25]. Therefore, the main goals of this study were to quantify the expression levels of the Bt toxins in the pollen of two transgenic cotton cultivars throughout the entire season and to determine the lethal and sublethal effects of the pollen on *A. mellifera* and *B. mori*. Li et al. measured the distribution of cotton pollen deposition and predicted the highest average pollen density to be 61.67 grains/cm^2^ at a distance of 0 m and 95.67 grains/cm^2^ at a distance of 1 m from the edge of the cotton field [35]. Based on the density of cotton pollen deposited naturally on leaves of mulberry plants and considering that silkworms can not survive independently in the field, we conducted a series of laboratory bioassays to determine the effects of Bt cotton pollen on *B. mori.*

## Materials and Methods

### Ethics Statement

All necessary permits were obtained for the described study, which complied with all relevant regulations. All Bt cotton cultivars were planted in the experimental field at Huazhong Agricultural University, Wuhan, China, and the University gave permission to conduct the study at this site. The field studies did not involve endangered or protected species.

### Pollen Collection

The two transgenic Bt cotton cultivars ZMSJ (expressing Cry1Ac/Cry2Ab) and ZMKCKC (expressing Cry1Ac/EPSPS) used in this study were gifts from the Institute of Cotton Research, the Chinese Academy of Agricultural Science. The local cotton variety, Emian 24 (non-GM cotton), was a gift from the National Key Laboratory of Crop Genetic Improvement, Huazhong Agricultural University. The ZMSJ cotton expresses two Bt proteins for the control of lepidopteran pests, such as the cotton bollworm *Helicoverpa armigera*. The ZMKCKC cotton expresses one gene for insect resistance and one gene for herbicide tolerance.

All cultivars were cultivated under recommended agronomic practices at the experiment field at Huazhong Agricultural University in early May 2011 without exposure to any pesticide. Pollen samples of each cultivar were collected using the multi-point field sampling method [18] on June 20^th^, July 20^th^, and August 20^th^ (early bloom, mid-stage bloom and late bloom respectively). The freshly collected cotton pollen samples were sieved (830 µm mesh size) and stored at –80°C until they were used for experiments or analyses.

### ELISA Quantitative Detection of Bt Proteins in Pollen

The quantities of Cry1Ac and Cry2Ab in each pollen sample were estimated using Envirologix Qualiplate Kits (EnviroLogix Quantiplate Kit, Portland, ME, USA). The detection limits for the two proteins were 0.1 ng/g and 0.52 ng/g, respectively. Before analysis, the fresh pollen samples were homogenized in 4 ml of extraction buffer and then kept at 4°C overnight for extraction of insecticidal proteins. After being centrifuged for 15 min at 7000 g, the supernatants of the extraction were used for the analyses.

### Experimental Insects and Treatment Applications

Worker bees of *A. mellifera* were obtained from the apiary of Huazhong Agriculture University. Bees were fed with sucrose solution daily and colonies were not treated with insecticides. Emerging honey bee adults (0 d) were collected from a colony during summer for bioassays.

The silkworm we used is a hybrid of *B. mori*, Qiufeng × Baiyu, which is the main variety used for commercial cocoon production in Southern China. Silkworm eggs were placed in an incubator set at 25±0.5°C and 75±5% relative humidity for hatching, and newly hatched larvae (neonates) were used in the bioassays.

For honey bees, feeding behavior was evaluated following the protocols described by Han et al. [18]. Emerging honey bees were kept in cages (15 × 10 × 20 cm) [36] with the top face covered with a piece of mesh, and they were used for the experiments after a 1-day period of adaptation to rearing conditions. Conventional cotton pollen, ZMSJ cotton pollen, and ZMKCKC cotton pollen were used in the experiments as three different treatments; Bt cotton pollen samples collected in July were used because they contained the highest amount of Bt toxin (see Table 1). Three different diets were prepared by mixing water, honey, and pollen at a ratio of 1∶2∶7 (weight) with no additional sugar provided. Five replicates (cage) were used per treatment with 40 bees per replicate, and during the bioassay process the honey bee mortality and pollen consumption were recorded daily. Honey bees were considered dead when they remained completely immobile, and they were removed from the cages every day [26]. After being exposed to the three different dietary treatments for 7 days, the surviving bees were prepared for the total hemocyte count (THC) experiment, in which 30 bees per treatment (five cages × six bees) were used. THC (number/µl) was determined using a phase contrast microscope (40×) with a hemocytometer [37].

**Table 1:** Cry1Ac and Cry2Ab protein content in cotton pollen from the transgenic ZMSJ cotton, ZMKCKC cotton and the non-Bt cotton as assayed by ELISA method.

Transgene proteins	Cotton variety	Contents of transgene proteins ± SD (ng/g fresh pollen)		
		Jun.20	Jul.20	Aug.20
Cry1Ac	ZMSJ	159.0±29.2b	572.5±28.1a	58.5±38.8c
	ZMKCKC	175.7±48.6b	544.5±22.5a	485.0±39.6a
	Non-Bt	0	0	0
Cry2Ab	ZMSJ	92.0±22.0a	92.4±23.1a	77.2±17.4a
	ZMKCKC	0	0	0
	Non-Bt	0	0	0

Values with the different letters are significantly different at the P<0.05 level (ANOVA followed by Tukey’s post-hoc test).

For silkworms, experiments were performed following the protocols described by Li et al. with slight modification [38]. Based on the density of cotton pollen deposited naturally on leaves of mulberry plants [35] and Hansen’s study [39], two different densities of each type of Bt cotton pollen and conventional cotton pollen were obtained by suspending 10 and 100 mg of pollen in 1 ml distilled water. For Bt pollen, we used samples collected in 20^th^ July. Based on the ELISA results in Table 1, the content of Bt toxins was calculated and the data were shown in Table 2. Fresh mulberry leaves were collected from the Mulberry Experiment Garden at Huazhong Agricultural University, which is situated far from the cotton fields. Leaf disks were cut using a 7.0 cm^2^-hole puncher and then dipped in the pollen suspension; the discs and suspension were shaken to ensure uniform distribution of pollen grains on the leaf surface. Under the microscope, the mean number of pollen grains on the leaves treated with 10 and 100 mg/ml pollen suspensions was approximately 900 and 8000 pollen grains/cm^2^, respectively. A non-pollen treatment, in which leaf disks were treated only with distilled water, served as the negative control. Each treatment was replicated six times with 10 neonates each time. Larvae were fed with treated leaves from birth to pupation. Both developmental phase and mortality were monitored for all individuals every day until pupation, and the weight of molting larvae (molters) for 1^st^ to 4^th^ instars was also measured. To evaluate the hemocyte concentration, another six replicates were used for each treatment with 10 neonates per replicate. Hemolymph was collected from 5^th^ instar larvae on days 1 (V-1), 3 (V-3), 5 (V-5), and 7 (V-7), and THC (number/µl) was determined using a blood cell counter as described by Tu et al. [40]. We use six insects for each THC test.

**Table 2:** Cry1Ac and Cry2Ab protein content in different food types of the silkworm *Bombyx mori.*

Pollen	Density(mg/ml)	Contents of transgene proteins ± SD (ng/ml)	
		Cry1Ac	Cry2Ab
ZMSJ	100	57.3±2.8	9.2±2.3
	10	5.7±0.3	0.9±0.2
ZMKCKC	100	54.5±2.3	0
	10	5.4±0.2	0
Non-Bt	100	0	0
	10	0	0
Control	0	0	0

### Data Analysis

The Cry proteins (Cry1Ac and Cry2Ab) content in cotton pollen was compared among the treatments using one-way analysis of variance (ANOVA) followed by Tukey’s post-hoc test. The data from honey bees were analyzed with mixed models and used replicate (cage) as a random factor. The survival dynamics of honey bees were analyzed with Cox proportional hazards regression models, and the cumulative pollen consumption and THC results for honey bees were fitted to a log-linear model.

The survival response of *B. mori* to different dietary treatments was analyzed using the Kaplan-Meier procedure and Logrank test. Nonparametric tests (K independent samples: Kruskal-Wallis H-tests; two independent samples: Mann-Whitney U tests) were performed on the developmental duration of *B. mori* larvae (from 1^st^ instar to 5^th^ instar), because the assumptions for parametric analyses were not fulfilled. The molter weight and THC results of *B. mori* larvae were compared using ANOVA, and means were compared by Tukey’s post-hoc test. All statistical tests were conducted using SAS Version 8.0 (SAS Institute Inc., Cary, NC, USA).

## Results

### ELISA Results for Cry1Ac and Cry2Ab in Cotton Pollens

The quantities of Cry1Ac or Cry2Ab in pollens of the two Bt cotton varieties were measured during the anthesis period from early bloom to late bloom. As expected, no Cry1Ac or Cry2Ab was detected in the non-Bt cotton. The amount of Cry2Ab protein in ZMSJ pollen was statistically steady throughout the season (all P>0.05). The highest amount of Cry1Ac protein in ZMSJ pollen was detected at mid-flowering, and the quantity was significantly lower in the early and late flowering periods (both P<0.001) (Table 1). For the ZMKCKC pollen, higher amounts of Cry1Ac protein were detected during mid and late bloom (with no difference between them, P = 0.13), whereas the quantity was significantly lower in the early bloom period (both P<0.001).

### Effect of Bt Pollen on Honey Bees

After 7 days, more than 70% of honey bees had survived in the treatments with Cry proteins and the control treatment, and no significant differences were detected between survival in the Bt pollen treatments and the control groups (χ^2^ = 0.71, df = 2, P = 0.70) (Fig. 1).

**Figure 1:** Survival analysis of honey bees from groups subjected to chronic exposure to ZMSJ pollen, ZMKCKC pollen and non-Bt pollen after 7 days. Data were analyzed with Cox proportional hazards regression models, and no significant differences were found among all the treatments at the P>0.05 level.

Cumulative consumption of pollen values were 28.4±2.2 mg for ZMSJ, 28.0±1.2 mg for ZMKCKC, and 32.5±2.6 mg for control, and no difference between the non-Bt and Bt pollen treatments was found (‘food type’ factor: χ^2^ = 2.11, df = 2, P = 0.35) (Table 3). The ‘replicate’ factor and its interaction with the ‘food type’ factor were not significant (replicate factor: χ^2^ = 0.47, df = 4, P = 0.98; and food type × replicate: χ^2^ = 1.21, df = 8, P = 0.99), meaning that different replicates had consistent results within the same food type.

**Table 3:** Cumulative consumption of pollen by honey bees from groups subjected to chronic exposure to ZMSJ pollen, ZMKCKC pollen and non-Bt pollen after 7 days.

Treatment			Cumulative consumption of pollen per bee ± SD (mg)
ZMSJ			28.4±2.2
ZMKCKC			28.0±1.2
Control			32.5±2.6
**Source of variation**	**df**	**χ^2^**	**P value**
Food type	2	2.11	0.35
Replicate	4	0.47	0.98
Food type × replicate	8	1.21	0.99

Statistics from the log linear model used to analyze the cumulative consumption of honey bees at the end of the oral chronic exposure period among treatments (food type factor) and as function of replicate factor.

Table 4 shows the THC of bees after exposure to Bt pollen for 7 days. No significant difference was found among all the treatments (‘food type’ factor: χ^2^ = 1.43, df = 2, P = 0.49). The ‘replicate’ factor and its interaction with the ‘food type’ factor were not significant (replicate factor: χ^2^ = 1.03, df = 4, P = 0.90; and food type × replicate: χ^2^ = 3.79, df = 8, P = 0.88), which indicates that, for the same food type, THC results were consistent among the different replicates.

**Table 4:** Mean total hemocyte count of honey bees from groups subjected to chronic exposure to ZMSJ pollen, ZMKCKC pollen and non-Bt pollen after 7 days.

Treatment			Total hemocyte count ± SD (µl)
ZMSJ			600.0±63.5
ZMKCKC			571.7±24.0
Control			545.0±46.7
**Source of variation**	**df**	**χ^2^**	**P value**
Food type	2	1.43	0.49
Replicate	4	1.03	0.90
Food type × replicate	8	3.79	0.88

Statistics from the log linear model used to analyze the total hemocyte count of honey bees at the end of the oral chronic exposure period among treatments (food type factor) and as function of replicate factor (five replicates per food type with six individual bees per replicate).

### Effect of Bt Pollen on Silkworms

Survivorship decreased from 96.7 to 76.7% across the whole larval period (the 1^st^ to the 5^th^ instar) among all treatments, and no statistical difference was observed in the survivorship for young larvae exposed to the two Bt pollen types, the non-Bt pollen, and the control diets (χ^2^ = 3.40, df = 6, P = 0.76) (Fig. 2).

**Figure 2:** Survival analysis of silkworm larvae treated with different doses of Bt-pollen or non-Bt pollen. No significant differences in survival rates were found among all the treatments at the P>0.05 level (followed by Kaplan–Meier survival analysis).

No significant difference in duration of developmental phase among treatments was found for the first two instars and fully matured larvae (Kruskal-Wallis H-test; 1^st^ instar: χ^2^ = 6.87, df = 6, P = 0.33; 2^nd^ instar: χ^2^ = 9.44, df = 6, P = 0.15; 5^th^ instar: χ^2^ = 6.78, df = 6, P = 0.34). For the 3^rd^ larval stage, larvae of *B. mori* fed the control diet had a significantly shorter developmental phase compared to those fed a high density of ZMSJ and ZMKCKC pollen (Mann-Whitney U test: P<0.001 and P = 0.04), or non-Bt pollen (P<0.001). In addition, 4^th^ instar *B. mori* larvae fed the control diet also had a significantly shorter developmental phase compared to those fed a high density of Bt and non-Bt pollen (all P<0.001). However, no difference was found between Bt and non-Bt pollen treatments at different pollen densities for the 3^rd^ and 4^th^ larval stages (all P>0.05) (Fig. 3).

**Figure 3:** Duration of development of silkworm larvae treated with different doses of Bt pollen or non-Bt pollen. Values with the different letter are significantly different. Bars represent standard error. Levels of significance: P<0.05 (followed by nonparametric tests-K independent samples: Kruskal-Wallis H-tests; two independent samples: Mann-Whitney U tests).

Total body weight of the molters was recorded and the weight distributions of the molters in the Bt pollen, non-Bt pollen, and control diet groups did not differ significantly after the first and final molting (1^st^ instar: F_6,385_ = 2.08, P = 0.055; 4^th^ instar: F_6,346_ = 1.36, P = 0.229). Just after the second and third moulting, larvae treated with high pollen density showed significant differences compared to the control (2^nd^ instar: F_6,367_ = 8.49, P<0.001; 3^rd^ instar: F_6,352_ = 7.99, P<0.001), but weights of Bt pollen fed larvae were almost identical to those of non-Bt pollen fed larvae (Fig. 4).

**Figure 4:** Weight of silkworm molters treated with different doses of Bt pollen or non-Bt pollen. A∼D represents the molter weight of the 1^st^ to 4^th^ instar larvae. Values with the different letter are significantly different. Bars represent standard error. Levels of significance: P<0.05 (ANOVA followed by Tukey’s post-hoc test).

When we evaluated the THC of the 5^th^ instar larvae, the results indicated that the hemocyte concentration increased with growth in the early and middle fifth instar phases and subsequently decreased during the prepupal stage (V-7). There were no significant differences in the THC of the V-1 and V-7 larvae among different treatments (V-1: F_6,35_ = 1.62, P = 0.172; V-7: F_6,35_ = 1.02, P = 0.428). THC of the V-3 larvae reared on ZMSJ pollen at the two different densities was significantly higher than that of the control, but differences between other pollen treatments and the control were not found (V-3: F_6,35_ = 17.76, P<0.001). For the V-5 larvae, the hemocyte concentration was significantly higher than that of the control only in the high density of ZMSJ and non-Bt pollen treatments (V-5: F_6,35_ = 18.04, P<0.001), and no significant differences were observed between Bt and non-Bt treatments (Fig. 5).

**Figure 5:** Mean total hemocyte count of silkworm treated with different doses of Bt pollen or non-Bt pollen. V-1, 3, 5, 7 represent the 1^st^, 3^rd^, 5^th^ and 7^th^ day of 5^th^ instar larvae. Bars represent standard error. Values with the different letter are significantly different at the P<0.05 level (ANOVA followed by Tukey’s post-hoc test).

## Discussion

In order to minimize the environmental risks of cultivating GM crops, it is necessary to identify the possible adverse effects of transgenic cotton on non-target species during their development, especially for economically important insects in China. Our study is, to the best of our knowledge, the first to evaluate the effects of stacked Bt cotton on *B. mori*.

### ELISA Results for Cry1Ac and Cry2Ab in Pollen

Knowing the concentration of toxic proteins expressed in pollen from transgenic cotton is very important for assessing its adverse impact on non-target insects [41]. It is crucial to identify a reliable expression level of insecticidal toxins in target GM crop tissues before conducting risk assessment because this value greatly impacts the effects on tested organisms [32]. The expression levels of transgenic proteins in the pollen of ZMSJ and ZMKCKC have not been reported previously.

In our study, the expression level of Cry1Ac in both Bt pollens varied greatly throughout the season, with the highest values in samples collected in July. This shows the importance of assessing toxin levels throughout the season. The level of the Cry2Ab toxin, however, was stable. Recent studies conducted on another GM cotton cultivar also demonstrated temporal variances in Cry1Ac protein expression [18], [25], [42].

### Effects of Pollen from Single and Multiple Bt Cotton Varieties on Honey Bees

One future trend in plant biotechnology is the stacking of multiple resistance traits in a single cultivar [13]. Honey bees are exposed to mass flowering GM crops, which contain multiple toxins or resistance traits, but only a few studies have examined the effect of stacked Bt crop on bees [13], [43]. Adverse effects of stacked transgenic cotton pollen on the survival, cumulative consumption, and THC of *A. mellifera* were not detected in this study. These findings suggest that the tested Bt cotton pollens have no deleterious effects on honey bees.

Neither larval nor adult honey bees have ever shown lethality when exposed to Bt proteins [44], [45], and our data also suggest that synergistic effects of stacking Bt proteins at plant-produced levels are unlikely a be a risk to emerging adult bees. At a realistic exposure dose, the 7 day survivorship of Bt-pollen treated bees in our study was similar to that of bees exposed to the conventional cotton pollen (Fig. 1). The results are in line with recent tests on Cry1Ac/CpTI cotton pollen [18], [41], [46], stacked Bt maize pollen [43] or purified Bt proteins [44], [45].

However, sublethal effects of the Bt pollen on larval development, feeding, learning performance, and foraging behavior might occur [13], [27], [37], [47]. Honey bee larvae and young adults (less than 12 days old) mainly feed on pollen [48], and nurse bees consume 3.4 to 4.3 mg of pollen per day [49]. Therefore, the potential risks of GM crop pollen on feeding behavior of *A. mellifera* needed to be assessed. In our study, after 7 days of chronic exposure to two stacked Bt pollens, no feeding inhibition occurred. Similar results were reported for studies of single [27], [47] or stacked Bt corn pollen [43]. Nevertheless, Han et al. reported an anti-feeding effect of Cry1Ac/CpTI cotton on honey bees [18]. However, that cultivar contained a different insect-resistant gene than the cultivar used in our study. Comparing Cry1 with transgenic protease inhibitors in many studies, only the latter impacted the feeding behavior [50]–[53]. Better knowledge about the sublethal risks associated with ZMSJ and ZMKCKC pollen for honey bees may also be obtained studying the effects of pollen [13] or multiple Bt proteins [45] on larval development.

In pollinators, information about potential sublethal physiological effects is scarce [54]. However, such effects could impact important biological processes, notably immunity. Honey bees defend themselves from an especially diverse range of pathogens, including bacteria, fungi, viruses, nematodes, protozoa, mites, flies, and beetles [55], [56]. Thus, it is important to determine if Bt toxins cause an immune reaction in honey bees. In this study, we assessed the risks of Bt cotton on the cellular immunity of honey bees. Higher THC is expected to be associated with higher resistance to disease [57]. Compared to the control, we found no negative effect of exposure to Bt pollen on THC in honey bees, which suggests that Bt pollens have no direct impact on honey bee health. This result is in line with a recent study that showed that most Cry proteins (>98%) in the bee gut were degraded, and had no harmful physiological effects on honey nurse bees [43].

### Effects of Pollen from Single and Multiple Bt Cotton Varieties on Silkworm

We found that exposure of *B. mori* larvae to different densities of pollen from either Bt cotton cultivar expressing Cry1Ac and Cry2Ab proteins had no adverse effects on young larval survival or development. This finding is consistent with results for pollens from Bt corn [23], [38] and rice [22]. Conversely, a transgenic Chinese cabbage pollen expressing Cry1Ac toxin adversely affected *B. mori* larvae when consumed [28]. Several factors may explain the differences in the response of *B. mori* to Bt pollens in different studies. For example, different pollens contain different levels of Cry protein levels. Furthermore, subspecies can vary in their susceptibility to Cry proteins [22].

Considering the importance of the insect hemocyte in the recognition and defense against microorganisms, we measured THC levels in 5^th^ instar *B. mori* larvae. At day 3 (V-3), the hemocyte concentration of larvae in the Cry1Ac/Cry2Ab cotton pollen treatment was increased relative to the control, indicating that the Cry1Ac/Cry2Ab cotton pollen caused an immune reaction. At day 5 (V-5), the high-density Cry1Ac/Cry2Ab cotton pollen treatment also had a significant influence on the immune system of *B. mori* larvae. However, in our experiments, the average density of cotton pollen deposited on mulberry leaves (approximately 900 and 8000 pollen grains/cm^2^) is much higher than that occurs under normal field conditions (<200 grains/cm^2^) [35], which indicates that the risk for *B. mori* was minimal. At day 7 (V-7, the day before larvae reached the pupal stage) there was no significant difference, showing that the pollen had no direct impact on the health of the preceding larval stages of *B. mori*.

Many factors affect the probability that *B. mori* larvae will be exposed to Bt cotton pollen. First, the cotton pollen density load on mulberry leaves is very important. The average density of cotton pollen naturally deposited on mulberry leaves [35] is lower than that of corn [38] or rice [22] pollen at the same distance from the edge of field. Under normal field conditions, the highest average cotton pollen density is 61.67 grains/cm^2^ at a distance of 0 m and 95.67 grains/cm^2^ at a distance of 1 m from the edge of the cotton field [35]. In our experiments, the mean number of pollen grains on the leaves treated with 10 and 100 mg/ml pollen suspensions was approximately 900 and 8000 pollen grains/cm^2^, which is substantially higher than the density that occurs under normal field conditions. Even in this worst-case feeding scenario, the Bt cotton pollen had little effect on the *B. mori* larvae.

Other important factors that can affect the impact of Bt pollen on non-target organisms are the degrees of hazard and exposure [51], [52]. The hazard posed by Bt cotton pollen to *B. mori* primarily depends on the type of Cry gene present. The insecticidal crystal proteins (ICPs) that are encoded by the Cry1Ac and Cry2Ab genes have specific activity against certain lepidopterans larvae, and both have been used in many GM crops [8], [53]. However, the mechanisms that underlie the specificity of these genes remain unclear. For example, Cry1Aa, Cry1Ab and Cry1Ac are all Cry1 genes, but Cry1Aa exhibits 400-fold greater toxicity against *B. mori* than Cry1Ac [22], [58]. Thus, it is likely that the transgenic products of the Cry1Ac and Cry2Ab genes in our tested Bt cottons have low toxicity against *B. mori.*

The low concentration of the Bt proteins to which *B. mori* larvae were exposed may have led to minimal effect observed, even at a very high pollen density. Several factors affect the level of exposure, but it is mainly related to the expression level of the proteins. In our study, the expression of Cry2Ab was far lower than that of Cry1Ac (Table 1), which was mainly due to the promoter used in transformation. Therefore, in the development of transgenic crops, a suitable promoter should be selected to ensure that the gene is highly expressed in the tissues attacked by target pests and expressed at lower levels in the pollen [22]. The amount of Cry1Ac and Cry2Ab proteins released from the ingested pollens to the larval midgut may also be an important factor that affects exposure to the toxic proteins in Bt pollen. Yao et al. showed that the digestibility rate of pollen grains in the digestive tract of *B. mori* is very low (less than 30%) [22], which suggests that the pollen from Bt cotton poses little risk to silkworms even if it contains high levels of toxic Bt proteins. Considering all of these factors, the adverse effects of pollen from Bt cottons on the survival, development, and hemocyte concentration of the silkworm appear to be minimal.

In summary, our data indicate that consumption of Bt cotton pollens expressing Cry1Ac and Cry2Ab did not negatively affect young adult *A. mellifera* or *B. mori* larvae. However, further experiments are underway to determine whether sublethal effects could impact later silkworm generations or the honey bee queen. In addition, the susceptibility of silkworm larvae of other varieties to the pollen should be evaluated, as different varieties of silkworm may have different susceptibilities to Bt insecticidal proteins. Field studies of honey bees also need to be conducted, as such studies are the most direct way to assess the potential impacts of planting Bt cotton on a commercial scale on non-target organisms [27].
